The article "Involvement of FOXO Transcription Factors, TRAIL-FasL/Fas, and Sirtuin Proteins Family in Canine Coronavirus Type II-Induced Apoptosis" was retracted in 2025. Reasons: plagiarized images; duplicated images; overlap with other authors' work; overlap with earlier publications.

# Involvement of FOXO Transcription Factors, TRAIL-FasL/Fas, and Sirtuin Proteins Family in Canine Coronavirus Type II-Induced Apoptosis

**DOI:** 10.1371/journal.pone.0027313

**Published:** 2011-11-08

**Authors:** Gabriella Marfè, Marco Tafani, Filomena Fiorito, Ugo Pagnini, Giuseppe Iovane, Luisa De Martino

**Affiliations:** 1 Department of Experimental Medicine and Biochemical Sciences, University of Rome “Tor Vergata”, Rome, Italy; 2 Department of Cellular and Molecular Pathology, IRCCS San Raffaele Pisana, Rome, Italy; 3 Department of Pathology and Animal Health, University of Naples “Federico II”, Naples, Italy; Yale Medical School, United States of America

## Abstract

n our previous study, we have shown that canine coronavirus type II (CCoV-II) activates both extrinsic and intrinsic apoptotic pathway in a canine fibrosarcoma cell line (A-72 cells). Herein we investigated the role of Sirtuin and Forkhead box O (FOXO) families in this experimental model using Nortern Blot and Western Blot analysis. Our results demonstrated that mitochondrial SIRT3 and SIRT4 protein expression increased from 12 and 24 h post infection (p.i.) onwards, respectively, whereas the nuclear SIRT1 expression increased during the first 12 h p.i. followed by a decrease after 36 h p.i., reaching the same level of control at 48 h p.i. Sirtuins interact with/and regulate the activity of FOXO family proteins, and we herein observed that FOXO3A and FOXO1 expression increased significantly and stably from 12 h p.i. onwards. In addition, CCoV-II induces a remarkable increase in the expression of TNF-related apoptosis-inducing ligand (TRAIL), while we observed a slight up-regulation of FasL/Fas at 36 p.i. with a decrease of both proteins at the end of infection**.** Furthermore, we found that virus infection increased both bax translocation into mitochondria and decreased bcl-2 expression in cytosol in a time-dependent manner.

These data suggest that FOXO transcription factors mediate pro-apoptotic effects of CCoV-II, in part due to activation of extrinsic apoptosis pathway, while some Sirtuin family members (such as SIRT3 and SIRT4) may be involved in intrinsic apoptotic pathway. Moreover, these results propose that TRAIL is an important mediator of cell death induced by CCoV-II during *in vitro* infection.

## Introduction

Canine coronavirus (CCoV), a member of antigenic group 1 of the family *Coronaviridae*, is a single positive-stranded RNA virus responsible for enteric disease in young puppies [1]. Two genotypes of CCoVs, CCoV-I and –II, have been described [2] sharing about 90% sequence identity in most of their genome, and CCoV-II is the only one which grows in cell cultures [2]. It has been shown that infection of a canine fibrosarcoma cell line (A-72 cells) by CCoV-II resulted in an apoptotic process [3], [4], depending on the activation of both intrinsic and extrinsic pathways of the caspases cascade but did not affect CCoV replication [4].

The article "Involvement of FOXO Transcription Factors, TRAIL-FasL/Fas, and Sirtuin Proteins Family in Canine Coronavirus Type II-Induced Apoptosis" was retracted in 2025. Reasons: plagiarized images; duplicated images; overlap with other authors' work; overlap with earlier publications.

Sirtuin proteins (SIRTs) are highly conserved nicotinamide adenine dinucleotide (NAD)-dependent histone deacetylases (HDACs) and constitute a recently identified mammalian family of regulatory molecules modulating the organism life span in many species [5]. Furthermore, they have been implicated in the control of critical cellular processes such as differentiation, proliferation, metabolism, senescence, apoptosis, as well as in transcriptional silencing, genetic control of aging, and calorie restriction-mediated longevity of organisms ranging from yeasts to humans [6], [7]. In mammals, there are seven members of the Sirtuin family of proteins (SIRT1 to SIRT7). Among those, SIRT1 also known as the guardian of cellular integrity, is primarily located in the nucleus. In addition to histones, SIRT1 has been shown to deacetylate other proteins, including forkhead transcription factors box O (FOXO) [8]. SIRT1 can monitor cellular metabolism and exert corresponding effects on gene expression. Previous studies showed that SIRT1 is a key regulator of cell defenses and survival in response to stress [8], and deacetylates and represses FOXO1 dependent apoptosis [9]. Other authors reported that SIRT1 increases the ability of FOXO3A to induce cell cycle arrest and resistance to oxidative stress, but inhibited the ability of FOXO3A to induce cell death [10]. In addition, FOXO transcription factors control cell proliferation and survival by regulating the expression of genes involved in cell-cycle progression, for instance cyclin D1/2, and apoptosis, for instance Bim, tumour-necrosis-factor-related apoptosis inducing ligand (TRAIL) and Fas ligand (FasL) [11], [12]. Cellular death receptors (DRs) transmit apoptosis-inducing signals initiated by specific death ligands, most of which are primarily expressed as biologically active type II membrane proteins that are cleaved into soluble forms. FasL activates Fas, and TRAIL activates DR4 (TRAILR1) and DR5 (TRAILR2) [13]. Moreover, TRAIL can activate the apoptotic pathway of cells by modulating the Bcl-2 family proteins, particularly the proapoptotic member Bax [14].

Although, SIRT1 represents the best-studied sirtuin, several studies have been published regarding others sirtuin proteins such as SIRT3, SIRT4 and SIRT5 [15]. The role of SIRT3 in the mechanisms of cell death and cell survival is still controversial. In fact, it has been demonstrated that the mitochondrial NAD-dependent deacetylase SIRT3 plays a role in the maintenance of basal ATP levels and as regulator of mitochondrial electron transport [16]. SIRT3 decreases mitochondrial membrane potential and reactive oxygen species production, while increasing cellular respiration [17]. Furthermore, SIRT3 regulates acetyl-CoA synthetase 2 [18], [19] and glutamate dehydrogenase [20], [21]. On the other hand, SIRT4 has been shown to inhibit glutamate dehydrogenase in pancreatic beta cells [15] and, in concert with SIRT3, to function as a mitochondrial NAD(+)-dependent deacetylase [22]. In this regards, it is important to note that little else is known about biological functions of SIRT4 [21]. Moreover, sirtuins also regulate viral transcription. SIRT1-SIRT3 can deacetylate the human immunodeficiency virus (HIV) 1 transactivator Tat, thereby promoting viral transcription [23]. Interestingly, the observation that SIRT1 inhibitors can reduce HIV transcription suggests that SIRT1 antagonists could prove useful to combat viral infection.

The article "Involvement of FOXO Transcription Factors, TRAIL-FasL/Fas, and Sirtuin Proteins Family in Canine Coronavirus Type II-Induced Apoptosis" was retracted in 2025. Reasons: plagiarized images; duplicated images; overlap with other authors' work; overlap with earlier publications.

The aim of the present study was to analyze the modulations of Sirtuin and FOXO family proteins during CCoV-II infection in a canine fibrosarcoma cell line (A-72 cells). We also investigated TRAIL and FasL/Fas pathways which are direct targets of FOXO transcription factor. Furthermore, in order to gain more insight into the intrinsic pathway, we studied the localization of both sirtuins (SIRT3 and SIRT4) and apoptotic proteins (bax and bcl-2) during the infection.

## Materials and Methods

### Cells and virus

A canine fibrosarcoma cell line (A-72 cells) (CRL-1542, American Type Culture Collection) was grown and maintained in complete medium consisting of Dulbecco Minimal Essential Medium (D-MEM) supplemented with 2 mM L-glutamine, 1% non essential amino acid, 5% heat-inactivated foetal calf serum (FCS), 100 IU of penicillin, and 100 µg of streptomycin per ml, at 37°C in a 5% CO_2_ atmosphere incubator. This cell line was maintained free of mycoplasma and of bovine viral diarrhoea virus. Cells were trypsinized once a week.

CCoV type II strain S/378 (kindly provided by Prof. C. Buonavoglia, Faculty of Veterinary Medicine, University of Bari, Italy) was used for the study. For viral infection A-72 cells at 80 to 90% confluence in complete medium as described above, were incubated with virus at multiplicity of infection (MOI) of 10. One hour post-infection (p.i.) non internalized virus was removed by washing the cells three times with DMEM, followed by incubation in complete medium. Virus titers were determined by end point dilution tests using 96-well microtitre plates, and are given as 50% tissue culture infective doses (TCID_50_) according to the method of Reed and Muench [24]. Aliquots of CCoV-II were stored at -80°C until used.

The article "Involvement of FOXO Transcription Factors, TRAIL-FasL/Fas, and Sirtuin Proteins Family in Canine Coronavirus Type II-Induced Apoptosis" was retracted in 2025. Reasons: plagiarized images; duplicated images; overlap with other authors' work; overlap with earlier publications.

### RNA isolation and Northern blot analysis

Total RNAs from mock-infected and infected cells at MOI 10 at different times p.i. were isolated using Tri Reagent (Sigma-Aldrich Chemie GmbH, Taufkirchen, Germany). Aliquots of RNA were electrophoresed on 1% agarose formaldehyde gels and subsequently blotted onto nylon membranes (Hybond N, Amersham, Braunschweig, Germany). The membrane was then UV crosslinked, and hybridized to ^32^P-labeled probe. Northern blot analysis is still a standard technique used in the detection and quantification of mRNA levels because it allows a direct comparison of the mRNA abundance between samples on a single membrane [25]. The relative amount of mRNA level was quantified throughout Gel-Doc Phosphorimanger and Quantity One software (Bio-Rad) and normalized by the band intensity of β-actin.

### Protein extraction and Western blot analysis

Mock-infected and infected cells (MOI 10) were collected at different times p.i. (4, 8, 12, 24, 36 and 48 h) and washed twice in PBS, then the cell pellets were homogenized directly into lysis buffer (50 mM HEPES, 150 mM NaCl, 1 mM EDTA, 1 mM EGTA, 10% glycerol, 1% NP-40, 1 mM phenylmethylsulfonyl fluoride, 1 µg/ml aprotinin, 0.5 mM sodium orthovanadate, and 20 mM sodium pyrophosphate). Lysates were centrifugated at 14,000×rpm for 10 min. Protein concentrations were determined by the Bradford assay (Bio-Rad, Hercules, CA). Equivalent amounts of proteins were loaded and electrophoresed on SDS-polyacrylamide gels. Subsequently, proteins were transferred to nitrocellulose membranes (Immobilon, Millipore Corp., Bedford, MA). After blocking with Tris-buffered saline-BSA (25 mM Tris (pH 7.4), 200 mM NaCl, and 5% BSA), the membrane was incubated with the following primary antibodies: anti-SIRT1 PAb (dilution 1∶1,500) (Everest Biotech Ltd), anti-SIRT3 PAb (dilution 1∶1,500) (Aviva Systems Biology), anti-SIRT4 PAb (dilution 1∶2,000) (Everest Biotech Ltd), anti-FOXO1 PAb (dilution 1∶1,500) (Aviva Systems Biology), anti-FOXO3A PAb (dilution 1∶1,500) (Aviva Systems Biology), anti-bax PAb (1∶1,000) (Aviva Systems Biology), anti-bcl-2 PAb (1∶1,000) (Abcam), anti-TRAIL MAb (1∶1000) (Cell Signaling), anti-FasL PAb (1∶1000) (Cell Signaling) anti-Fas PAb (1∶1000) (Abcam), anti-TIM50 PAb (1∶2000) (Everest Biotech Ltd) and anti-β-actin MAb (dilution 1∶7,500) (Cell Signaling). Membranes were then incubated with the appropriate horseradish peroxidase-conjugated secondary antibody (dilution 1∶1,000) (at room temperature), and the reaction was detected with an enhanced chemiluminescence system (Amersham Life Science). The relative amount of protein expression was quantified using Gel-Doc phosphorimanger and Quantity One software (Bio-Rad) and normalized by the band intensity of β-actin or TIM50.

The article "Involvement of FOXO Transcription Factors, TRAIL-FasL/Fas, and Sirtuin Proteins Family in Canine Coronavirus Type II-Induced Apoptosis" was retracted in 2025. Reasons: plagiarized images; duplicated images; overlap with other authors' work; overlap with earlier publications.

### Cytosolic and mitochondrial protein extraction

Isolation of mitochondria and cytosolic fractions were carried out using a modified protocol from Kluck et al. [26]. Mock-infected and infected cells were collected at different times p.i. and washed twice in PBS. The cell pellets were resuspended in lysis buffer (50 mM Tris [pH 7.5], 150 mM NaCl_2_, 5 mM EGTA, 1 mM CaCl_2_, 1 mM MgCl_2_, 1% NP-40, 1 µg/ml leupeptin, 1 µg/ml aprotinin, 1 µM PMSF, and 100 µM Na_3_VO_4_). Samples were then incubated on ice for 20 minutes and centrifuged at 14,000 rpm for 15 min to obtain the cytosolic fraction in the surnatant. The pellet (mitochondria-enriched fraction) was resuspended in the mitochondrial buffer (70 mM Tris base, 0.25 M sucrose and 1 mM EDTA, pH 7.4). Equivalent amounts of proteins were loaded and electrophoresed on SDS-polyacrylamide gels. The Western blot analysis was performed, as reported above. The relative amount of protein expression was quantified using Gel-Doc phosphorimanger and Quantity One software (Bio-Rad) and normalized by the band intensity of β-actin or TIM50.

### **RNA isolation and** Semi-quantitative RT-PCR analysis

Total RNAs were isolated using Tri Reagent. One microgram of total RNA from each samples was transcribed with Superscript II Reverse Transcriptase reverse transcriptase^c^ at 37°C for 60 min with the final stage at 90°C for 5 min. PCR was carried out on cDNA using a Stratagene RoboCycler Gradient 40 temperature cycler fitted with a Hot Top Assembly, using 500 µl thin-walled PCR tubes. The primers, designed with the Primer3 program, are listed below:

SIRT1

sense 5’-TGGAAAGTCCGGATTTGAAG-3’’

antisense 5-AGCGCCATGGAAAATGTAAC-3’

SIRT3

sense 5’-GGCCTGAGGAAGAGTGTGAG-3’’

antisense 5-GCAGATTCAGTCTGGGCTTC-3’

SIRT4

sense 5’-GCTTTGAGCAACTGGGAAAG-3’

antisense 5’-CAAAGGACCCTGAAACCAAA-3’

FOXO3A

sense 5’-GCAAGCACAGAGTTGGATGA-3’

antisense 5’-CAGGTCGTCCATGAGGTTTT-3’

FOXO1

sense 5’-AAGAGCGTGCCCTACTTCAA-3’

antisense 5’-CTGTTGTTGTCCATGGATGC-3’.

The conditions for PCR amplification of cDNA were as follows: one cycle at 95°C for 5 min as an initial denaturation step; then, denaturation at 95°C for 30 sec, annealing at 58°C (SIRT1, SIRT3, SIRT4, FOXO3A and FOXO1) and 60°C (β-actin) for 30 sec, and extension at 72°C for 90 sec, followed by further incubation for 15 min at 72°C (1 cycle). After 40 cycles (β-actin) [27], 35 cycles (SIRT1, SIRT3, SIRT4, FOXO3A, FOXO1), shown to be at the linear phase of amplification, the PCR products were electrophoresed onto a 1.6% agarose gel.

The article "Involvement of FOXO Transcription Factors, TRAIL-FasL/Fas, and Sirtuin Proteins Family in Canine Coronavirus Type II-Induced Apoptosis" was retracted in 2025. Reasons: plagiarized images; duplicated images; overlap with other authors' work; overlap with earlier publications.

Densitometry and band quantization was performed using BioRad Quantity One software.

### Statistical analysis

The results are presented as mean ± SEM of three experiments. One-way ANOVA with Tukey's post test was performed using GraphPad InStat Version 3.00 for Windows 95 (GraphPad Software, San Diego, CA, USA). P value <0.05 was considered statistically significant.

## Results

### Gene regulation of members of Sirtuin, FOXO and Bcl-2 families during CCoV-II-induced apoptosis

The SIRT1, SIRT3, SIRT4, FOXO3A, FOXO1, bax and bcl-2 mRNA expression levels were evaluated by Northern blot analysis on total RNA extracted at different times during CCoV-II infection. The level of SIRT1 mRNA showed a significant increase (P<0.001) at 12, 24 and 36 h p.i., reaching about the same level of control at 48 h p.i. (Figure 1A, B). FOXO3A and FOXO1 mRNA content increased significantly (P<0.001) and their values remained higher up to 48 h p.i. (Figure 1A, B). Furthermore, we found that the SIRT3 transcript levels increased from 12 h p.i. (P<0.01) with the rise becoming more significant later in the infection (P<0.01; P<0.001) (Figure 2A, B), while SIRT4 transcript levels increased at 12 h p.i. (P<0.01) and remained constant at this higher level until the end of infection (Figure 2A, C). In addition, the levels of bax mRNA were observed to be similar when compared to those of control cells during the first hours p.i., but we observed at 12 h p.i. a significant increase (P<0.001) which did not change until the end of infection (Figure 3A, B). Whereas, the level of bcl-2 mRNA showed a significant decrease from 12 h p.i onwards (P<0.001) (Figure 3A, B).

**Figure 1:** CCoV-II infection modulates the gene regulation of SIRT1, FOXO3A, FOXO1, mRNA level. (**A**) To perform Northern blot assay, RNA was extracted from mock-infected (lanes cc, control cells) and infected cells at the indicated times, electrophoresed and hybridized with a labelled probe as described under Material and Methods. β-actin was used as loading control. Blot is representative of three separate experiments. (**B**) Densitometric analysis of blots relative to SIRT1, FOXO3A, FOXO1 (panel B). The bars represent the mean ± SEM of the results from three separate experiments. Significant differences between CCoV-II-infected cells and control cells are indicated by probability *P*. ***P <0.001.

**Figure 2:** CCoV-II infection modulates the gene regulation of SIRT3 and SIRT4. (**A**) To perform Northern blot assay, RNA was extracted from mock-infected (lanes cc, control cells) and infected cells at the indicated times, electrophoresed and hybridized with a labelled probe as described under Material and Methods. β-actin was used as loading control. Blot is representative of three separate experiments. (**B**) Densitometric analysis of blots relative to SIRT3. The bars represent the mean ± SEM of the results from three separate experiments. Significant differences between CCoV-II-infected cells and control cells are indicated by probability *P*. **P <0.01, and ***P <0.001. (**C**) Densitometric analysis of blots relative to SIRT4. The bars represent the mean ± SEM of the results from three separate experiments. Significant differences between CCoV-II-infected cells and control cells are indicated by probability *P*. **P <0.01.

The article "Involvement of FOXO Transcription Factors, TRAIL-FasL/Fas, and Sirtuin Proteins Family in Canine Coronavirus Type II-Induced Apoptosis" was retracted in 2025. Reasons: plagiarized images; duplicated images; overlap with other authors' work; overlap with earlier publications.

**Figure 3:** CCoV-II infection modulates the gene regulation of bax and bcl-2. (**A**) To perform Northern blot assay, RNA was extracted from mock-infected (lanes cc, control cells) and infected cells at the indicated times, electrophoresed and hybridized with a labelled probe as described under Material and Methods. β-actin was used as loading control. Blot is representative of three separate experiments. (**B**) Densitometric analysis of blots relative to bax and bcl-2. The bars represent the mean ± SEM of the results from three separate experiments. Significant differences between CCoV-II-infected cells and control cells are indicated by probability *P*. ***P <0.001.

### Protein expression of TRAIL, Sirtuin and FOXO families members during CCoV-II-induced apoptosis

In order to better understand the interaction between SIRT1 and FOXO family during the CCoV-II-induced apoptosis, we performed Western blot analysis. As shown in Figure 4A and B, we observed a different expression pattern of SIRT1, FOXO3A and FOXO1. In particular, significant increases of SIRT1, FOXO3A and FOXO1 protein levels were evident at 12 h p.i. (P<0.01) (Figure 4A, B). Expression levels of SIRT1 protein peaked at 12 h p.i. The levels of SIRT1 were significantly higher than control levels at 24 (P<0.05), and 36 h p.i. (P<0.05) and although they had dropped by 48 h p.i. they were not significantly lower than those of the control (Figure 4A, B). Whereas, the trend of FOXO3A expression level presented a significant increase at 24 (P<0.01), 36 (P<0.001) and at 48 h p.i. (P<0.05) (Figure 4A, B). Instead, the increase of FOXO1 expression level occurred from 12 h p.i. (P<0.01) but the expression level of FOXO1 becomes more significant at 24, 36 and 48 h p.i. (P<0.001) (Figure 4A, B). We next examined the effect of virus on the protein expression of TRAIL, FasL and Fas, which are direct targets of FOXO transcription factors. Following infection, TRAIL expression levels were significantly enhanced from 12 h p.i. (P<0.01), reaching a peak at 36 h p.i. (P<0.001) (Figure 5A, B), when we also detected a slight but significant increase (P<0.05) of FasL/Fas (Figure 6A, B, C). However, at the end of infection, we observed a significant decrease in FasL protein expression levels (P<0.01) compared to mock infected cells (Figure 6A, B).

The article "Involvement of FOXO Transcription Factors, TRAIL-FasL/Fas, and Sirtuin Proteins Family in Canine Coronavirus Type II-Induced Apoptosis" was retracted in 2025. Reasons: plagiarized images; duplicated images; overlap with other authors' work; overlap with earlier publications.

**Figure 4:** CCoV-II infection modulates the SIRT1, FOXO3 and FOXO1 proteins expression. (**A**) Whole-cell lysates were prepared from mock-infected (lanes cc, control cells) and infected cells at the indicated times. Western blot analysis was performed with antibodies specifically recognizing SIRT1, FOXO3A and FOXO1. β-actin was used as an internal loading control. The molecular weight (in KDa) of protein size standards is shown on the left hand side. Blot is representative of three separate experiments. (**B**) Densitometric analysis of blots relative to SIRT1, FOXO3A and FOXO1. The bars represent the mean ± SEM of the results from three separate experiments. Significant differences between CCoV-II-infected cells and control cells are indicated by probability *P*. *P <0.05, **P <0.01, and ***P <0.001.

**Figure 5:** CCoV-II infection modulates TRAIL protein expression. (**A**) Cell lysates were collected at the indicated times p.i., and equal amounts of proteins from each sample were subjected to Western blot analysis and probed for TRAIL antibody which recognized the 28–30 KDa bands for TRAIL-R1 and TRAIL-R2, respectively. β-actin was used as a loading control. The molecular weight (KDa) of protein size standards is shown on the left hand side. Blot is representative of three separate experiments. (**B**) Densitometric analysis of blots relative to TRAIL 30 and TRAIL 28. The bars represent the mean ± SEM of the results from three separate experiments. Significant differences between CCoV-II-infected cells and control cells are indicated by probability *P*. **P <0.01, and ***P <0.001.

**Figure 6:** CCoV-II infection modulates FasL/Fas proteins expression. (**A**) Cell lysates were collected at the indicated times p.i., and equal amounts of proteins from each sample were subjected to Western blot analysis and probed for FasL and Fas. β-actin was used as a loading control. The molecular weight (KDa) of protein size standards is shown on the left hand side. Blot is representative of three separate experiments. (**B**) Densitometric analysis of blots relative to FasL and (**C**) Fas. The bars represent the mean ± SEM of the results from three separate experiments. Significant differences between CCoV-II-infected cells and control cells are indicated by probability *P*. *P <0.05 and **P <0.01.

In order to better characterize the mitochondrial pathway, we evaluated protein expression levels of SIRT3 and SIRT4 in the mitochondrial and cytosolic fractions. Both SIRT3 and SIRT4 were detected only in the mitochondrial fraction where SIRT3 started to increase significantly at 12 h p.i. (P<0.001) (Figure 7A, B), while SIRT4 only from 24 h p.i. onwards (P<0.001; P<0.01) (Figure 8A, B).

The article "Involvement of FOXO Transcription Factors, TRAIL-FasL/Fas, and Sirtuin Proteins Family in Canine Coronavirus Type II-Induced Apoptosis" was retracted in 2025. Reasons: plagiarized images; duplicated images; overlap with other authors' work; overlap with earlier publications.

**Figure 7:** CCoV-II infection modulates SIRT3 protein expression in mitochondrial fraction. (**A**) Cell lysates were collected at the indicated times p.i., and equal amounts of proteins from each sample were subjected to Western blot analysis and probed for SIRT3. TIM50 was used as a loading control. The molecular weight (KDa) of protein size standards is shown on the left hand side. Blot is representative of three separate experiments. (**B**) Densitometric analysis of blots relative to SIRT3. The bars represent the mean ± SEM of the results from three separate experiments. Significant differences between CCoV-II-infected cells and control cells are indicated by probability *P*. *P <0.05, **P <0.01, and ***P <0.001.

**Figure 8:** CCoV-II infection modulates SIRT4 protein expression in mitochondrial fraction. (**A**) Cell lysates were collected at the indicated times p.i., and equal amounts of proteins from each sample were subjected to Western blot analysis and probed for SIRT4. TIM50 was used as a loading control. The molecular weight (KDa) of protein size standards is shown on the left hand side. Blot is representative of three separate experiments. (**B**) Densitometric analysis of blots relative to SIRT4. The bars represent the mean ± SEM of the results from three separate experiments. Significant differences between CCoV-II-infected cells and control cells are indicated by probability *P*. **P <0.01 and ***P <0.001.

### Intracellular localization of bax and bcl-2 in CCoV-II-induced apoptosis

In order to validate both the results obtained by SIRT3, SIRT4 and TRAIL Western blots, we determined also bax and bcl-2 protein expression in the cytosolic and mitochondrial fractions during the infection. As shown in Figure 9A and B, the expression of pro-apoptotic member bax significantly decreased in the cytosolic fraction from 12 h p.i. onwards (P<0.01, P<0.001), whereas, in the mitochondrial fraction, significantly increased at the same times (P<0.001), indicating the translocation of this protein from the cytosol into the mitochondrial compartment following infection (Figure 9A, B). By contrast, the expression of the anti-apoptotic protein bcl-2, was detected only in the cytosolic fraction where it decreased significantly (P<0.01, P<0.001) in a time-dependent manner during infection (Figure 9A, C).

The article "Involvement of FOXO Transcription Factors, TRAIL-FasL/Fas, and Sirtuin Proteins Family in Canine Coronavirus Type II-Induced Apoptosis" was retracted in 2025. Reasons: plagiarized images; duplicated images; overlap with other authors' work; overlap with earlier publications.

**Figure 9:** CCoV-II infection induces bax translocation into the mitochondria and bcl-2 decrease. (**A**) A-72 cells were mock-infected (lane cc, control cells) and CCoV-II infected (4, 8, 12, 24, 36 and 48 h p.i.). The bax and bcl-2 expression was evaluated in the cytosol and in the mitochondrial fractions during the infection; equal amounts of proteins from each sample were subjected to Western blot analysis and probed for bax and bcl-2. β-actin and TIM50 were used as a loading control. The molecular weight (KDa) of protein size standards is shown on the left hand side. Blot is representative of three separate experiments. (**B**) Densitometric analysis of bax and (**C**) of bcl-2 are shown below the blots. The bars represent the mean ± SEM of the results from three separate experiments. Significant differences between CCoV-II-infected cells and control cells are indicated by probability *P*. **P <0.01 and ***P <0.001.

### Semi-quantitative RT-PCR analysis of Sirtuin and FOXO proteins families

Semi-quantitative RT-PCR analysis of key proteins, herein examined, confirmed the results above reported. In fact, from 12 h p.i. onwards, generally we detected a significant increase of SIRT1, SIRT3, SIRT4 as shown in Figure 10 (P<0.01, P<0.001), and of FOXO3A, FOXO1 as shown in Figure 11 (P<0.01, P<0.001).

**Figure 10:** Expression of SIRT1, SIRT3 and SIRT4 cDNA of mock-infected and infected cells at the indicated times at different post infection. (**A**) The RT-PCR products were examined by 1.6% agarose gel electrophoresis. (**B**) Densitometric analysis of the corresponding band to SIRT1, SIRT3 and SIRT4. The bars represent the mean ± SEM of the results from three separate experiments. Significant differences between CCoV-II-infected cells and control cells are indicated by probability *P*. **P <0.01 and ***P <0.001.

**Figure 11:** Expression of FOXO3A and FOXO1 cDNA of mock-infected and infected cells at the indicated times at different post infection. (**A**) The RT-PCR products were examined by 1.6% agarose gel electrophoresis. (**B**) Densitometric analysis of the corresponding band to FOXO3A and FOXO1. The bars represent the mean ± SEM of the results from three separate experiments. Significant differences between CCoV-II-infected cells and control cells are indicated by probability *P*. **P <0.01 and ***P <0.001.

## Discussion

Sirtuins are considered key regulators of cell survival and apoptosis through their interaction with nuclear and mitochondrial proteins. Moreover, it is established that sirtuins interact with and regulate the activity of FOXO gene family proteins [28], [29]. Since SIRT1 itself does not bind to DNA directly, targeted deacetylation of histones is thought to occur through its interaction with specific DNA binding factors, such as FOXO3A and FOXO1. Thus, SIRT1 can bind and deacetylate FOXO3A and FOXO1, leading to a selective augmentation of FOXO-regulated stress resistance genes [9], [10]. In this study, to better understand the mechanism of canine coronavirus type II-induced apoptosis, we examined the role of SIRT1, SIRT3 and SIRT4 during the CCoV-II infection. Furthermore, we investigated the evolving relationship between SIRT1 and FOXO3A/FOXO1 members. Our data show a different pattern in both gene and protein expression of SIRT1, FOXO3A and FOXO1 over the course of CCoV-II infection. After an early up-regulation of SIRT1, we observed after 12 h p.i. a gradual decrease in expression when levels fell back to those of the control cells. Such modification in expression level of SIRT1 might led to an increased expression of pro-apoptotic FOXO targets such as bim. This hypothesis is consistent with our previous work in which we have observed an increased time-dependent expression of bim during the CCoV-II infection [4]. On the other hand, it was already reported that the FOXO3A/FOXO1-induced cell death is mediated through bim, which is one of the FOXO-target genes [30]-[32]. It has also been shown that expression levels of TRAIL, FasL and Fas, which are further transcriptional targets of FOXO, can control cell cycle and apoptosis [31], [33]–[37]. For this reason, in the present study, we also investigated protein expression of TRAIL, FasL and Fas. In our study, it appears that TRAIL expression level increased at 12 h p.i., when CCoV-II-induced apoptosis starts, as previously described [4]. While a slight up-regulation in the expression of FasL/Fas protein levels occurred only in the late stage of infection. Our results suggest that CCoV-II infection modulates the TRAIL expression levels more than that of FasL/Fas, suggesting that the contribution of TRAIL with respect to that of FasL/Fas is more crucial in CCoV-II-induced extrinsic apoptotic pathway. Strong induction of TRAIL but not FasL expression in SARS coronavirus infected human monocytes derived dendritic cells was also observed [38]. In general, viral infection can lead to apoptosis of host cells, through two apoptotic pathways, the death receptors pathway (extrinsic pathway) and the mitochondrion pathway (intrinsic pathway). These two pathways interact together to coordinate apoptosis [39]. Particularly, infection of a canine fibrosarcoma cell line by CCoV-II resulted in an apoptotic process [3], [4] depending on the activation of both intrinsic and extrinsic pathways of the caspases cascade [4]. Previously, we demonstrated that CCoV-II triggers apoptosis in A-72 cells through the release of cytochrome *c* from mitochondria, and alterations in the pro- and anti-apoptotic members of Bcl-2 family [4]. To better understand the mitochondrial alterations, herein, we have also examined the role of some mitochondrial SIRT proteins. It is known that the coordinated actions of two mitochondrial sirtuins, SIRT3 and SIRT4, are able to inhibit cell death by maintaining constant mitochondrial NAD^+^ levels following stress [22]. In this study, we observed the SIRT3 and SIRT4 increase in the mitochondria depending upon CCoV-II-infection. Recently, it has been shown that SIRT3 can block bax translocation to the mitochondria and hence prevent cardiomyocytes stress-mediated cell death [40]. Since we observed an increasing trend of SIRT3 expression from 12 p.i. onwards, such result could either suggest that, in our system, SIRT3 does not render infected cells resistant to bax-mediated cell damage or, more likely, that SIRT3 facilitates the apoptotic pathway activated by CCoV-II. In fact, SIRT3 has been associated with induction of cell death by regulating distinct basal apoptotic pathways [41] and SIRT3 overexpression has also been shown to increase in kaempferol induced apoptosis [42]. The increasing trend of SIRT4 in the mitochondria with peaks at 24 and 36 hours of post infection that we observed is more difficult to interpret due to the fact that very little is known about the activity and specificity of SIRT4 in apoptosis.

The article "Involvement of FOXO Transcription Factors, TRAIL-FasL/Fas, and Sirtuin Proteins Family in Canine Coronavirus Type II-Induced Apoptosis" was retracted in 2025. Reasons: plagiarized images; duplicated images; overlap with other authors' work; overlap with earlier publications.

Furthermore, we also considered bax and bcl-2 expression levels in the cytosolic and mitochondrial fractions. We present evidence that the pro-apoptotic protein bax translocates from the cytosol to the mitochondrial compartment, while the antiapoptotic protein Bcl-2 was down-regulated in the cytosolic compartment. Our data show that this apoptotic pathway induces the positive modulation of bax/bcl-2 ratio, in which TRAIL can be involved.

In conclusion, our results support the notion that the up-regulation of TRAIL may be a primary mediator of CCoV-II-induced apoptosis, and that the mitochondrion plays a critical role in a host defense mechanism showing an involvement of SIRT (precisely SIRT3 and SIRT4) and FOXO families proteins in this infection, in part due to activation of both extrinsic and intrinsic apoptosis pathway. The link between activation of the FOXO proteins and cell death was well established, and it was identified the role of the pro-apoptotic gene FasL in the activation of the death receptor Fas/CD95/APO-1 promoting mitochondria-independent apoptosis [11], [12]. For this reason, we believe that both the activation of extrinsic apoptotic pathway by FOXO transcription factors, TRAIL-FasL/Fas, and the activation of intrinsic apoptotic pathway by Sirtuin proteins such as SIRT3 and SIRT4 occurred during CCoV-II infection.

The article "Involvement of FOXO Transcription Factors, TRAIL-FasL/Fas, and Sirtuin Proteins Family in Canine Coronavirus Type II-Induced Apoptosis" was retracted in 2025. Reasons: plagiarized images; duplicated images; overlap with other authors' work; overlap with earlier publications.

To our knowledge, no investigation has so far been carried out about SIRT and FOXO families proteins involvement on other viral infection.
